The article "Efficacy and Mechanism of Mallotus furetianus Müll. Arg. Extract on Nonalcoholic Fatty Liver Disease" was published in 2022. Journal: Evid Based Complement Alternat Med.

# Efficacy and Mechanism of *Mallotus furetianus* Müll. Arg. Extract on Nonalcoholic Fatty Liver Disease

**DOI:** 10.1155/2022/4897463

**Published:** 2022-04-28

**Authors:** Daobin Lin, Yi Ding, Yabo Cheng, Yubin Chen, Yunting Tang, Xiaowen Wu, Yawei Cheng

**Affiliations:** ^1^Department of Cardiology, Hainan Provincial Hospital of Traditional Chinese Medicine, Haikou 570293, China; ^2^Department of Disease Prevention, Hainan Provincial Hospital of Traditional Chinese Medicine, Haikou 570293, China; ^3^Department of Wrist, Sichuan Orthopedic Hospital, Chengdu 610041, China; ^4^Department of Disease Prevention, Hainan Hospital of Traditional Chinese Medicine Affiliated to Guangzhou University of Chinese Medicine, Haikou 570100, China

## Abstract

Nonalcoholic fatty liver disease (NAFLD) is currently the major cause of chronic liver disease globally. To observe the sedative effect of *Mallotus furetianus* extract (MFE) on NAFLD and the potential molecular mechanism, a high-fat diet (HFD) was used to induce NAFLD in rats for 8 weeks. Rats were orally given MFE (1.7 g/kg, 2.5 g/kg, and 3.3 g/kg) every day. Serum and liver biochemical indexes were detected. 16S rDNA sequencing was performed to test the changes in the gut microbiota. Mass spectrometry was used to analyze the changes in blood and liver metabolites and to perform a joint analysis of differential flora and differential metabolites. The results showed that MFE alleviated liver injury and decreased hepatic lipids content. ELISA analysis certificated that MFE reduced inflammation levels in rats fed with HFD. Compared to HFD rats with a normal diet, MFE significantly changed the overall structure of the intestinal flora and the composition of the intestinal microbes destroyed by HFD. In addition, MFE changes the metabolic levels of lipids and proteins in HFD rats. In conclusion, MFE effectively treated NAFLD and significantly improved the overall structure and intestinal microbial composition of the intestinal microbiota. The abundance of *Bacteroides fragilis* and *Escherichia coli* increased significantly in the partridge tea treatment group.

## 1. Introduction

NAFLD has now become an important cause of chronic liver disease in developed countries. The prevalence of NAFLD in adult people is 10% to 30%, of which 10% to 20% are nonalcoholic steatohepatitis (NASH). The incidence of liver cirrhosis is as high as 25% within 10 years [1, 2]. NAFLD covers many disease states, such as fatty liver, nonalcoholic steatohepatitis, fibrosis, cirrhosis, and hepatocellular carcinoma. Various levels of metabolic factors such as insulin resistance, dyslipidemia, and inflammation are increasingly regarded as the main pathogenic factors leading to liver steatosis, but the specific pathogenesis of NAFLD is complex and unclear [3, 4]. In addition, there is currently no approved treatment for NAFLD, so new treatments to treat this complex liver disease are urgently needed [3, 4].

The article "Efficacy and Mechanism of Mallotus furetianus Müll. Arg. Extract on Nonalcoholic Fatty Liver Disease" was published in 2022. Journal: Evid Based Complement Alternat Med.

*Mallotus furetiamus* is an economic plant from Hainan Island in China. Its leaves are used as an aromatic beverage and as a folk remedy for the treatment of cholecystitis [5]. The extract also has antioxidant and antiatherosclerotic activities. The water extract can reduce intracellular lipid accumulation in oleic acid-induced fat degeneration of liver cancer cells [5]. These results indicate that MF is effective in treating liver steatosis.

The intestinal flora has an important regulatory effect on NAFLD. The intestinal flora could affect the intestinal permeability, the luminal metabolism of cholecystic acid, lipoprotein lipase, endogenous alcohol, and toxic compounds [6, 7]. Increased intestinal permeability and lipoprotein lipase production in intestinal diseases contribute to the pathogenesis of NAFLD. The gut microbiota, which affects bile cholic acid biosynthesis in the course of NAFLD by regulating the liver-like protein X receptor (FXR) and HF-induced liver steatosis, inhibits the gut by changing the gut microbiota [8, 9]. The fermentation of short-chain fatty acids and carbohydrates produced by intestinal microorganisms helps to inhibit fat synthesis and accelerate the oxidation of fat in the liver. Some enzymes produced by gut microbes convert choline in food into toxic compounds, which are then absorbed by the liver, leading to liver damage and inflammation. In addition, the intestinal flora is the primary source of endogenous alcohol, and in patients with NASH. Large numbers of bacteria have been reported to produce alcohol [10–12]. Treatment with probiotics or prebiotics to relieve NAFLD is effective, further confirming the influence of intestinal flora on NAFLD. Therefore, regulating the intestinal flora is a potential treatment for NAFLD. In this study, HFD was used to induce NAFLD in rats, and 16S rDNA sequencing and metabolomics were used to analyze the regulatory effect and molecular mechanism of MFE on NAFLD.

## 2. Materials and Methods

### 2.1. Experimental Animals

Fifty male Wistar rats (200–250 g, 4–6 weeks old) were obtained from the Shanghai Laboratory Animal Center of Chinese Academy of Sciences (Shanghai, China). The animals were fed with standard laboratory feed and allowed to drink tap water at will. All animals were appropriately treated in accordance with the institutional animal care guidelines approved by the Experimental Animal Ethical Committee of Hainan Provincial Hospital of Traditional Chinese Medicine (IACUC-20200112-02).

The article "Efficacy and Mechanism of Mallotus furetianus Müll. Arg. Extract on Nonalcoholic Fatty Liver Disease" was published in 2022. Journal: Evid Based Complement Alternat Med.

### 2.2. Treatment of Rats

Fifty rats were divided into 5 groups randomly: normal-chow diet (NCD) (*n* = 10); HFD (*n* = 10); HFD + MFE (1.7 g/kg) (*n* = 10); HFD + MFE (2.5 g/kg) (*n* = 10); and HFD + MFE (3.3 g/kg) (*n* = 10). MFE is dissolved in physiological saline solution. The rats were fed HFD, and MFE was administered daily for 8 weeks.

### 2.3. Analysis of Serum ALT/AST Activities

The blood sample was stored at 4°C for 2 hours and then centrifuged at 860 xg for 15 minutes before serum collection. The kit was used to measure serum ALT and AST according to the manufacturer's instructions [10–12].

### 2.4. Assessment of IL-1*β*, IL-6, TNFa, and ADS/LEP

For each rat, commercial ELISA kits were utilized to quantify the level of serum tumor inflammatory factors (IL-1*β*, IL-6, and TNFa) and serum ADS/LEP, in accordance with the manufacturer's instructions [13].

### 2.5. Liver Histological Evaluation

Liver sections were fixed in 10% formalin solution for 24 hours and then embedded in paraffin. The specimen sections (5 *µ*m) were stained with hematoxylin-eosin (H&E) to observe the histology of liver damage. Oil red O staining was performed to observe the accumulation of lipids in the liver [14].

### 2.6. DNA Extraction, PCR Amplification, and MiSeq Sequencing

Samples were stored at −80°C until the DNA is extracted. QIAamp DNA Stool Mini Ki was used to extract all genomic DNA from each sample. As mentioned earlier, PCR amplification and MiSeq sequencing were performed. In summary, Phusion High-Fidelity PCR Master Mix and HF buffer (New England Biolabs, UK) were used to amplify the V4-V5 region of the bacterial 16S rDNA. Barcode index PCR primers 515F and 926R were used. The amplicon library with the AXYGEN AxyPrep DNA Gel Extraction Kit (AXYGEN Scientific, Union City, CA, USA) was purified, normalized with FTC-3000TM Real-Time PCR, using the MiSeq instrument (Illumina), using 2 × 300 cycles of V3 reagents. The cassette is sequenced.

### 2.7. Bioinformatics Analysis

The original sequencing reads were optimized, and bioinformatics analysis was performed. Simply put, the original data are demultiplexed according to the barcode. Trimmomatic (version 0.35) was used to eliminate poor-quality base pairs. FLASH (version 1.2.11) and mothur (version 1.33.3) were used to merge and filter the truncated reads. The multivariate statistical analysis was carried out with mothur, UPARSE (USEARCH version v8.1.1756), and R (version 3.2.3). The clean labels are aggregated in OTU and then assigned to the corresponding taxon according to the Silva 119 database. The multifactor analysis was performed to assess the total structural changes in the intestinal flora, and the sparse curve and alpha diversity were tested to assess the richness and diversity of each group of intestinal flora. The main coordinate analysis (PCoA) was performed based on the UniFrac distance and the UniFrac tree. mothur and R were used to analysis of *α*-diversity and *β*-diversity [15].

The article "Efficacy and Mechanism of Mallotus furetianus Müll. Arg. Extract on Nonalcoholic Fatty Liver Disease" was published in 2022. Journal: Evid Based Complement Alternat Med.

### 2.8. Metabolomic Analysis

A liquid chromatography (LC) quadrupole mass spectrometry (MS) amino acid analysis system with two independent liquid phase time-of-flight (LC-time) mass spectrometry platforms was used to measure the level of metabolites in the serum. For liver samples, the above 3 LC-MS platforms were analyzed by methanol/water extraction.

### 2.9. Statistical Analysis

Data are expressed as mean ± standard error of mean (SEM). Significant differences were determined by one-way analysis of variance (one-way ANOVA) and LSD post test. *P* < 0.05 was considered statistically significant.

## 3. Results

### 3.1. MFE Does Not Affect Weight in Rats Fed with HFD

After pathological examination confirmed that the model was successfully established, rats were given 1.7 g/(kg·d), 2.5 g/(kg·d), and 3.3 g/(kg·d) partridge tea solution by intragastric administration, and the normal group and the model group were given 10 ml/(kg·d) body weight distilled water orally. The administration period was 4 weeks, during which all rats were fed with basic feed and free drinking water, and weighed once a week.  Figure 1(a) shows the body weight curve from 0 to 12 weeks after treatment. No significant differences were found between the groups.  Figure 1(b) is the change in overall body weight within 12 weeks. It can be said that MFE has no effect on weight gain from a high-fat diet.

### 3.2. MFE Reduced Liver Injury in Rats Fed with HFD

As shown in Figures 2(a)–2(c), MFE (1.7, 2.5, and 3.3 g/kg) reduced the increased serum ALT, AST, and GGT activities induced by HFD in rats. Moreover, the effect of MFE (3.3 g/kg) was better than the other two doses. The liver H&E staining results indicated that MFE could reduce HFD-induced liver steatosis in rats (Figure 2(d)).

### 3.3. MFE Reduced Hepatic Lipids Accumulation in Rats Fed with HFD

The results showed that MFE (1.7, 2.5, and 3.3 g/kg) reduced the increased contents of serum TC, TG, LDL-C, and HDL-C induced by HFD in rats. In addition, the effect of 3.3 g/kg MFE was better than the other dose (Figure 3).

### 3.4. MFE Reduced Inflammation Levels in Rats Fed with HFD

Next, the expression of inflammation factors was detected in rats. The results showed that MFE (1.7, 2.5, and 3.3 g/kg) reduced the increased contents of serum IL-1*β*, IL-6, TNFa, LEP, and ADP induced by HFD in rats (Figure 4). Moreover, the effect of 3.3 g/kg MFE was better than the other dose.

The article "Efficacy and Mechanism of Mallotus furetianus Müll. Arg. Extract on Nonalcoholic Fatty Liver Disease" was published in 2022. Journal: Evid Based Complement Alternat Med.

### 3.5. MFE Changed the Composition of the Gut Microbiota

16S rDNA sequencing generated 593,121 high-quality sequences and 1,625 OTUs from 30 stool samples. Wien image analysis showed that the overall microbial diversity between the three groups was significantly different (Figure 5(a)). The dilution curve shows that the depth of the current sequence is sufficient and OTU is common (Figure 5(b)). According to the weighted and unweighted table of PCoA results, compared with the control group, the structure of the intestinal flora of the HFD group with the second major component (PC2) changed, and these changes were reversed after high-dose MFE administration (Figures 5(c) and 5(d)). Weighted and unweighted UniFrac trees show three different microbial communities in each group (Figures 5(e) and 5(f)).

In addition, LEfS was performed to analyze the statistical differences between the three groups. In the clade diagram, the circles radiating from the inside to the outside indicate the order level from the strain to the genus (or species). Each small circle of different degrees represented a level of the level, and the diameter of the small circle was proportional to the relative frequency. Species without a significant difference were colored yellow and biomarkers of different species were colored according to the group. The red knot represented the microbiome that plays an important role in the MFE group, and the green knot represented the microbiome that plays an important role in the MFE high-dose group. The blue knot represented the microbial taxa that play an important role in the NAFLD group (Figure 6(a)).

The LDA value distribution histogram showed species with an LDA score greater than 4, showing species with significant differences in abundance in different groups, and the length of the histogram represented the impact of different species (Figure 6(b)). Further analysis of the relative abundance of the biomarker in each group of samples found that *Bacteroides fragilis* and *Escherichia coli* in the NCD group were significantly higher than those in the other two groups, *Staphylococcus xylosus* in the MFE group was significantly higher than that in the other two groups, and *Ruminococcus flavefaciens* in the NAFLD group was significantly higher than the other two groups (Figure 6(c)). In addition, we combined the 16S flora analysis data with the metabolome. We found that the abundance of *Bacteroides* was negatively correlated with the contents of 3R, 6'Z)-3,4-dihydro-8-hydroxy-3-(6-pentadecenyl)-1H-2-benzopyran-1-one, 4,5-dihydropiperlonguminine, 8-hydroxypinoresinol 4-glucoside, cytidine, hypoxanthine, isoniazid alpha-ketoglutaric acid, L-isoleucine, and prolyl-alanine, and positively correlated with the contents of taurochenodesoxycholic acid, p-aminobenzoic acid, and marmesin rhamnoside (Figure 6(d)).

The article "Efficacy and Mechanism of Mallotus furetianus Müll. Arg. Extract on Nonalcoholic Fatty Liver Disease" was published in 2022. Journal: Evid Based Complement Alternat Med.

## 4. Discussion

In recent years, NAFLD has become more and more common in the world, which has attracted widespread attention from researchers and doctors [16]. Studies have shown that a variety of Chinese herbal medicines and natural active ingredients extract have good therapeutic prospects for NAFLD [17–19]. These studies provide new ideas for the treatment of NAFLD to find effective drugs from traditional Chinese medicine. MFE has a lipid-lowering effect and is widely used in the treatment of NAFLD [20]. MFE has a lipid-lowering effect on the blood and liver of rats with HFD fed [5]. HFD is widely used to induce experimental NAFLD in mice, and its pathology is very similar to human NAFLD [21]. In this study, liver TG, CT levels, and liver histopathology and staining showed that MFE reduced liver lipid accumulation in high-fat diet rats. These results further confirmed the protective effect of MFE on NAFLD and proved the great potential of MFE in the clinical treatment of NAFLD.

Elevated serum ALT and AST activities are usually signs of liver cell damage. Liver cell damage was related to the occurrence of NAFLD [22]. The results indicated that MFE also reduced the increased ALT/AST activity in the serum of HFD-fed rats, suggesting that it has a protective effect on liver cell damage during the progression of NAFLD. To determine the causes of weight loss and anti-inflammatory effects, we analyzed the gut microbiota of rats. The *α*-diversity analysis showed that the microbial accumulation of liraglutide in NAFLD rats was significantly reduced and not reversed. The *β*-diversity analysis shows that liraglutide has a significant influence on the composition of the intestinal flora. Hence, we speculate that liraglutide may have received a healthier composition of the intestinal flora, that is beneficial for lipid metabolism and inhibits inflammation.

Previous studies have shown that *Phascolarctobacterium*, *Blautia*, *Ruminococcus*, *Clostridium*, etc., in the samples of the NAFLD group are significantly increased, and they all have the ability to ferment to produce short-chain fatty acids (SCFAs) in the human intestine. Studies have shown that NAFLD affects the intestinal SCFA content. The level of SCFAs detected in the feces of NAFLD patients is increased, and the concentration of SCFAs produced by bacterial fermentation is relatively higher, suggesting a more adequate energy intake. The content of *Lachnospiraceae* in the NAFLD group was significantly reduced. *Lachnospiraceae* is a butyrate-producing bacteria. Its reduced content can significantly reduce the content of butyrate in SCFAs. Butyrate can be used as an important energy source for colon cells and also participates in inhibiting inflammation and enhanced screen long function. These indicate that the concentration of SCFAs in the intestinal tract of NAFLD is increased, which may only be due to the increase in the content of some of them, such as acetic acid [23]. We combined the 16S flora analysis data with the metabolome and found that the contents of (3R, 6'Z)-3,4-dihydro-8-hydroxy-3-(6-pentadecenyl)-1H-2-benzopyran-1-one, 4,5-dihydropiperlonguminine, 8-hydroxypinoresinol 4-glucoside, cytidine, hypoxanthine, isoniazid alpha-ketoglutaric acid, L-isoleucine, prolyl-alanine, taurochenodesoxycholic acid, p-aminobenzoic acid, and marmesin rhamnoside were correlated with the flora in the NAFLD group. This study is consistent with previous studies, showing that the intestinal flora can regulate metabolic pathways and participate in regulating the life activities of the body.

The article "Efficacy and Mechanism of Mallotus furetianus Müll. Arg. Extract on Nonalcoholic Fatty Liver Disease" was published in 2022. Journal: Evid Based Complement Alternat Med.

## 5. Conclusion

MFE reduced liver damage and lipid accumulation in NAFLD rats. MFE significantly improved the overall structure and intestinal microbial composition of the intestinal microbiota. The abundance of *Bacteroides fragilis* and *Escherichia coli* increased significantly in the MFE treatment group. In future research, we will further clarify the molecular regulation mechanism and target of MFE based on molecular docking, affinity chromatography, and coprecipitation experiments and lay a better research foundation for the clinical application of MFE.

## Figures and Tables

**Figure 1:** MFE does not affect weight in rats fed with HFD. (a) The body weight curve from 0 to 12 weeks after treatment (*n* = 7–9). (b) The change in overall body weight within 12 weeks. Data were expressed as mean ± SEM. ns, no significance.

**Figure 2:** MFE reduced liver injury in rats fed with HFD, with 10 rats in each group. (a) Detection of serum ALT activity. (b) Detection of serum AST activity. (c) Detection of serum GGT activity (*n* = 10). (d) Liver H&E staining. Magnification, 200 times. (I) NCD, (II) HFD, (III) HFD + MFE (1.7 g/kg), (IV) HFD + MFE (2.5 g/kg), and (V) HFD + MFE (3.3 g/kg). Data were expressed as mean ± SEM. ^#^*P* < 0.05, ^##^*P* < 0.01.

**Figure 3:** MFE reduced hepatic lipids accumulation in rats fed with HFD. (a) The content of serum TC (*n* = 10). (b) The content of serum TG (*n* = 10). (c) The content of serum LDL-C (*n* = 10). (d) Serum HDL-C (*n* = 10). Data were expressed as mean ± SEM. ^#^*P* < 0.05, ^##^*P* < 0.01.

The article "Efficacy and Mechanism of Mallotus furetianus Müll. Arg. Extract on Nonalcoholic Fatty Liver Disease" was published in 2022. Journal: Evid Based Complement Alternat Med.

**Figure 4:** MFE reduced inflammation levels in rats fed with HFD. (a) The content of serum IL-1*β* (*n* = 10). (b) The content of serum IL-6 (*n* = 10). (c) The content of serum TNFa (*n* = 10). (d) The content of serum LEP (*n* = 10). (e) The content of serum ADP (*n* = 10). Data were expressed as mean ± SEM. ^*∗*^*P* < 0.05, ^*∗∗*^*P* < 0.01.

**Figure 5:** *α*-Diversity analysis and structural changes of the gut microbiota. (a) Venn picture of multiple samples. (b) Rarefaction curves. (c) Weighted table of PCoA results. (d) Unweighted table of PCoA results. (e) Weighted UniFrac trees. (f) Unweighted UniFrac trees.

**Figure 6:** LEfSe analysis of the flora with statistical differences between the three groups. (a) Clade diagram. (b) Histogram. (c) The relative abundance of biomarker samples in each group. (d) Combined analysis of 16S flora analysis data and metabolome.

## Data Availability

The data used to support this research are included within this manuscript.
